# MicroRNA-216a inhibits the metastasis of gastric cancer cells by targeting JAK2/STAT3-mediated EMT process

This article has been retracted.

**DOI:** 10.18632/oncotarget.21488

**Published:** 2017-10-04

**Authors:** Youmao Tao, Songbai Yang, Yuanyu Wu, Xuedong Fang, Yannan Wang, Yan Song, Tao Han

**Affiliations:** ^1^ Department of Gastrointestinal Colorectal and Anal Surgery, China-Japan Union Hospital of Jilin University, Changchun, Jilin Province 130033, China; ^2^ Department of Vascular Surgery, China-Japan Union Hospital of Jilin University, Changchun, Jilin Province 130033, China

**Keywords:** miR-216a, tumor metastasis, gastric cancer, JAK2/STAT3, epithelial-mesenchymal transition

## Abstract

MicroRNAs (miRNAs), a group of small, non-protein coding, endogenous RNAs, play critical roles in the tumorigenesis and progression of human cancer. miR-216a has recently been reported to play an oncogenic role in human cancer. While, the expression of miR-216a, its biological function and underlying molecular mechanisms in gastric cancer (GC) are largely unknown. In this study, we revealed that miR-216a was underexpressed in GC tissues compared to matched noncancerous tissues. Decreased levels of miR-216a were confirmed in GC cell lines compared with a normal gastric epithelium cell line. miR-216a underexpression was associated with malignant prognostic features including lymph node metastasis, venous infiltration, invasive depth and advanced TNM stage. GC patients with low miR-216a level showed an obvious shorter overall survival. miR-216a overexpression restrained migration and invasion of MGC-803 cells, while its knockdown exerted opposite effects on metastatic behaviors of SGC-7901 cells. *In vivo* experiments found that miR-216a restoration reduced metastatic nodes of GC cells in nude mice liver. miR-216a notably suppressed epithelial-mesenchymal transition (EMT) of GC cells. Janus kinase 2 (JAK2) was recognized as a direct target and downstream mediator of miR-216a in GC cells. Interestingly, JAK2/signal transducer and activator of transcription 3 (STAT3) pathway was prominently inactivated by miR-216a and probably mediated the role of miR-216a in the regulation of migration, invasion and EMT process of GC cells. In conclusion, these data suggest that miR-216a functions as a tumor suppressive miRNA in the development of GC possibly by targeting JAK2/STAT3-mediated EMT.

## INTRODUCTION

Gastric cancer (GC) is known as the most common type of the malignant gastric tumor and one of the most deadly cancers worldwide [1]. The clinical outcome of GC patients is extremely poor [2], largely due to local and systemic metastasis of GC [3]. Several signaling pathways are implicated in metastasis of GC, such Janus kinase (JAK)-signal transducer and activator of transcription 3 (STAT3) and Notch signaling pathways [4, 5]. Recently, microRNAs (miRNAs) have been suggested as critical regulator of metastasis of GC [6, 7]. However, the mechanisms underlying metastasis of GC is still poorly investigated.

Increasing evidences support the role of miRNAs as tumor suppressors or oncogenes in human cancer. miRNAs are small, non-coding, single-stranded RNAs involved in post-translational regulation of gene expression and have been implicated in a wide range of essential biological activities [8]. Aberrant miRNA expression is strongly correlated with the development of metastasis in various cancers, including GC [9]. miR-216a has recently been reported to play a tumor suppressive role in human cancer including glioma [10], colorectal cancer (CRC)[11] and pancreatic cancer [12, 13]. miR-216a suppresses invasion, migration and proliferation of glioma cells by inhibiting leucine-rich repeat-containing G protein-coupled receptor 5 (LGR5)[10]. Furthermore, miR-216a prohibits invasion and migration of CRC cells *in vitro*, and restrains liver metastasis *in vivo* by targeting KIAA1199 [11]. miR-216a restrains pancreatic tumor growth via inducing G2/M arrest and apoptosis by decreasing lncRNA MALAT1 [12]. On the contrary, miR-216a facilitates epithelial-mesenchymal transition (EMT) of ovarian cancer cells and subsequently promotes migration and invasion of tumor cells [14]. miR-216a/217 overexpression induces EMT of hepatocellular carcinoma (HCC) cells and promotes recurrence and sorafenib resistance of HCC [15]. These studies suggest that the role of miR-216a is a controversial topic in different cancers. To date, the exact role of miR-216a in GC and its target genes are poorly elucidated.

In this study, we were aimed to investigate the expression and biological function of miR-216a in GC. We disclosed that the expression of miR-216a was restrained in GC. miR-216a inhibited migration, invasion and EMT process of GC cells probably by targeting JAK2/STAT3 pathway.

## RESULTS

### miR-216a expression is downregulated in GC tissues and cells

The expression of miR-216a was detected by qRT-PCR in GC and matched noncancerous tissues. miR-216a was found to be downregulated in GC tissues than in matched non-tumor tissues (P<0.05, Figure 1A). Subsequent study demonstrated that miR-216a expression was strongly reduced in GC cells (SGC-7901, MGC-803, MKN-28, and BGC-823 compared to GES-1 cells (P<0.05, respectively, Figure 1B). The “low” versus “high” miR-216a expression was defined according to the cut-off values of miR-216a level which were defined as the median of the cohort of tested patients. The clinicopathological significance of miR-216a expression in GC patients was shown in Table 1. Low level of miR-216a notably correlated with lymph node metastasis, venous infiltration, invasive depth and advanced TNM stage (P<0.05, respectively). In addition, GC patients with low miR-216a level showed a significant shorter survival (P<0.05, Figure 1C). Multivariate Cox regression analysis indicated that miR-216a expression was an independent risk factor for poor prognosis of GC patients (P=0.018, Table 2). Thus, miR-216a underexpression potentially functions as a predictor for poor prognosis of GC patients.

**Figure 1:** The expression and prognostic value of miR-216a in GC **(A)** The relative expressions of miR-216a in 90 pairs of GC tissues and matched noncancerous tissues. Data were presented as log2 of fold change of GC relative to matched noncancerous tissues and analyzed by student’s t-test. **(B)** qRT-PCR analysis of miR-216a expression in GC cell lines (SGC-7901, MGC-803, MKN-28, and BGC-823) and the normal human gastric epithelium cell line (GES-1). n = three repeats with similar results, ^*^P<0.05 by ANOVA. **(C)** GC patients were divided into miR-216a high expression group and miR-216a low expression group based on the median level of miR-216a expression. GC patients with low miR-216a level (n = 45) had an obvious shorter overall survival compared to those with high miR-216a level (n = 45). P<0.05 by Log-rank test.

**Table 1:** Association between the clinicopathological features and miR-216a expression in gastric cancer patients

Characteristics		n=90	miR-216a expression		*P*
			Low level (n=45)	High level (n=45)	
Age (y)	≤60	35	15	20	0.280
	>60	55	30	25	
Gender	Female	33	15	18	0.512
	Male	57	30	27	
Lymph node metastasis	Present	52	19	33	0.003^*^
	Absent	38	26	12	
Tumor size (cm)	≤5	24	13	11	0.634
	>5	66	32	34	
Venous infiltration	Present	39	14	25	0.019^*^
	Absent	51	31	20	
Invasive depth	T_1_	19	4	15	0.004^*^
	T_2_-T_4_	71	41	30	
Tumor differentiation	Well/Moderate	43	23	20	0.527
	Poor/Signet	47	22	25	
TNM stage	I+II	46	18	28	0.035^*^
	III+IV	44	27	17	

T1: mucosa (m), submucosal (sm); T2-T4: muscularis propria (mp), subserosa (ss), serosa exposed (se), serosa infiltrating (si). ^*^ Statistically significant.

**Table 2:** Multivariate Cox regression analysis of 5-year overall survival of gastric cancer patients (n=90)

Variables	Overall survival		
	HR	95% CI	*P*
Lymph node metastasis (present *vs* absent)	4.14	2.48-5.05	0.035^*^
Tumor size (cm, >5 *vs* ≤5)	1.46	0.92-1.88	0.091
Venous infiltration (present *vs* absent)	1.20	0.80-1.79	0.166
Invasive depth (T_2_-T_4_ *vs* T_1_)	2.05	1.41-2.60	0.007^*^
Tumor differentiation (poor/signet *vs* well/moderate poor)	1.37	0.82-1.86	0.364
TNM stage (III+IV *vs* I+II)	3.23	2.41-4.23	0.006^*^
miR-216a expression (low *vs* high)	2.12	1.51-2.50	0.018^*^

HR, hazard ratio; CI, confidence interval. ^*^Statistically significant.

### miR-216a inhibits migration and invasion of GC cells

Next, to determine the role of miR-216a in GC cells, we transfected MGC-803 cells with precursor miR-216a and scrambled controls (miR-control), respectively. miR-216a overexpression was confirmed by the qRT-PCR results (P<0.05, Figure 2A). Upon miR-216a restoration, MGC-803 cells showed significantly reduced migration and invasion compared to control cells (P<0.05, respectively, Figure 2B and 2C). On the other hand, miR-216a was knocked down by miR-216a inhibitors in SGC-7901 cells (P<0.05, Figure 2D). miR-216a knockdown promoted migration and invasion of SGC-7901 cells (P<0.05, respectively, Figure 2E and 2F). In addition, liver metastasis model showed that miR-216a overexpresion significantly reduced the number of metastatic nodules in livers arising from nude mice (P<0.05, Figure 3). Altogether, our data indicate that miR-216a plays an anti-metastatic role in GC cells.

**Figure 2:** miR-216a inhibits migration and invasion of GC cells **(A)** MGC-803 cells that were transfected with precursor miR-216a (pre-miR-216a) or scrambled controls (miR-control) were subjected to qRT-PCR for miR-216a expression. n = three repeats with similar results, ^*^P<0.05 by t test. **(B)** Wound healing assays indicated that miR-216a overexpression inhibited migration of MGC-803 cells. n = three repeats with similar results, ^*^P<0.05 by t test. **(C)** The number of invaded cells was reduced after miR-216a restoration in MGC-803 cells. n = three repeats with similar results, ^*^P<0.05 by t test. **(D)** SGC-7901 cells that were transfected with miR-216a inhibitors (anti-miR-216a) or scrambled controls (anti-control) were subjected to qRT-PCR for miR-216a expression. n = three repeats with similar results, ^*^P<0.05 by t test. **(E)** Wound healing assay indicated that miR-216a knockdown promoted migration of SGC-7901 cells. n = three repeats with similar results, ^*^P<0.05 by t test. **(F)** The number of invaded cells was increased after miR-216a loss in SGC-7901 cells. n = three repeats with similar results, ^*^P<0.05 by t test.

**Figure 3:** miR-216a suppresses liver metastasis of GC cells in mice MGC-803 cells that were transfected with precursor miR-216a (pre-miR-216a) or scrambled controls (miR-control) were intravenously injected into tail vein in nude mice. HE staining revealed that miR-216a overexpression significantly reduced the number of metastatic nodes of MGC-803 cells in nude mice livers. Scale bar: 1mm. n = 6, ^*^P<0.05 by t test.

### miR-216a suppresses EMT process of GC cells

To further explore the underlying mechanisms involved in the anti-metastatic role of miR-216a in GC cells, we aimed to investigate the regulatory effects of miR-216a on EMT, which was recognized as a main cause for cell migration and invasion. Interestingly, miR-216a overexpression led to increased expression E-cadherin and decreased levels of N-cadherin and Vimentin in MGC-803 cells (P<0.05, respectively, Figure 4A). IF results further confirmed the changes of E-cadherin and Vimentin expression after miR-216a restoration (Figure 4B). In turn, miR-216a knockdown facilitated EMT process of SGC-7901 cells with decreased E-cadherin and increased N-cadherin and Vimentin expression, as determined by immunoblotting and IF results (P<0.05, respectively, Figure 4C and 4D). These results indicate that miR-216a inversely regulates EMT process of GC cells.

**Figure 4:** miR-216a retrains EMT process of GC cells **(A)** MGC-803 cells that were transfected with precursor miR-216a (pre-miR-216a) or scrambled controls (miR-control) were subjected to immunoblotting for E-cadherin, N-cadherin and Vimentin expression. n = three repeats with similar results, ^*^P<0.05 by t test. **(B)** IF data revealed that miR-216a overexpression enhanced E-cadherin staining while reduced Vimentin staining in MGC-803 cells. **(C)** SGC-7901 cells that were transfected with miR-216a inhibitors (anti-miR-216a) or scrambled controls (anti-control) were subjected to immunoblotting for E-cadherin, N-cadherin and Vimentin expression. n = three repeats with similar results, ^*^P<0.05 by t test. **(D)** IF data revealed that miR-216a knockdown reduced E-cadherin staining while enhanced Vimentin staining in SGC-7901 cells.

### miR-216a directly targets JAK2 in GC cells

Potential targets of miR-216a were predicted using the public database TargetScan (http://www.targetscan.org), and the putative complementary sequence of miR-216a was identified in the 3′-UTR of JAK2 mRNA, as illustrated in Figure 5A. JAK2 mRNA and protein expression levels were determined after miR-216a overexpression. Our data showed that JAK2 expression was obviously downregulated by miR-216a overexpression in both MGC-803 and BGC-823 cells (P<0.05, respectively, Figure 5B and 5C). To further validate our hypothesis, we performed a luciferase reporter assay. As shown in Figure 5D, cells transfected with wt JAK2 3′-UTR vector containing a precursor miR-216a showed significantly lower luciferase activity than cells transfected with miR-control (P<0.05). In contrast, no changes in relative luciferase activity were observed when the miR-216a binding site was mutated (Figure 5D). Subsequently, Spearman correlation analysis revealed that JAK2 mRNA levels were negatively correlated with miR-216a levels in GC tissues (r=-0.529, P=0.006, Figure 5E). Representative IHC data showed that strong staining of JAK2 was observed in GC tissues with low miR-216a level, while weak signal of JAK2 was detected in cases with high miR-216a level (Figure 5F). Quantitative data suggested that the JAK2 expression in GC tissues with high miR-216 level was significantly decreased compared with those with low miR-216a level (P<0.05, Figure 5F). Based on these findings, we suggest that JAK2 is a potential direct target of miR-216a in GC cells.

**Figure 5:** JAK2 is a direct target of miR-216a in GC cells **(A)** The potential miR-216a binding site in wild type (wt) 3’-UTR sequence of JAK2. The underlined part is the mutant site designed for mutant (mt) 3’-UTR sequence of JAK2. **(B)** and **(C)** MGC-803 and BGC-823 cells that were transfected with precursor miR-216a (pre-miR-216a) or scrambled controls (miR-control) were confirmed by qRT-PCR and immunoblotting for JAK2 expression. n = three repeats with similar results, ^*^P<0.05 by t test. **(D)** miR-216a overexpression decreased the luciferase activity of wt 3’-UTR of JAK2. In contrast, no changes in relative luciferase activity were observed when the miR-216a binding site was mutated. n = three repeats with similar results, ^*^P<0.05 by t test. **(E)** An inverse correlation between the levels of JAK2 mRNA and miR-216a expression was observed in GC tissues. n = 90, P<0.05 by Spearman’s rank correlation test. **(F)** Representative IHC staining showed that miR-216a low expressing GC tissue (n = 45) showed strong staining of JAK2, while weak staining of JAK2 was observed in miR-216a high expressing case (n = 45). The JAK2 levels in high-miR-216a PADCs were significantly lower than that of those low-miR-216a GCs. Scale bar: 50μm. ^*^P<0.05 by t test.

### miR-216a inhibits migration and invasion of GC cells probably by targeting JAK2/STAT3 pathway

JAK2 is reported to be a upstream regulator of STAT3 [16]. Thus, we investigated the regulatory effects of miR-216a on activation of JAK2/STAT3 pathway in GC cells. Notably, miR-216a overexpression reduced the expression of phosphorylated STAT3 and its downstream targets including Slug, Snail and Twist in MGC-803 cells (P<0.05, respectively, Figure 6). In accordance, miR-216a knockdown promoted activation of JAK2/STAT3 pathway in SGC-7901 cells (P<0.05, respectively, Figure 6). Next, we disclosed whether JAK2 mediated the role of miR-216a in migration, invasion and EMT process of GC cells. We found that JAK2 restoration promoted the phosphorylation of STAT3 and EMT process, and subsequently facilitated migration and invasion of miR-216a overexpressing MGC-803 cells (P<0.05, respectively, Figure 7A-7C). Furthermore, the JAK2 inhibitor SAR317461 was used for inactivation of JAK2/STAT3 pathway in miR-216a down-regulating GC cells. SAR317461 treatment blocked JAK2/STAT3 pathway and suppressed migration, invasion and EMT process of SGC-7901 cells with miR-216a knockdown (P<0.05, respectively, Figure 8A-8C). Thus, miR-216a exerts its anti-metastatic role probably by targeting JAK2/STAT3 pathway in GC cells.

**Figure 6:** miR-216a inhibits activation of JAK2/STAT3 pathway MGC-803 cells that were transfected with precursor miR-216a (pre-miR-216a) or scrambled controls (miR-control) were detected by immunoblotting. miR-216a overexpression led to reduced levels of JAK2, phophorylated STAT3, Slug, Snail and Twist in MGC-803 cells. On the other hand, SGC-7901 cells that were transfected with miR-216a inhibitors (anti-miR-216a) or scrambled controls (anti-control) were subjected to immunoblotting. miR-216a knockdown promoted activation of JAK2/STAT3 pathway in SGC-7901 cells. n = three repeats with similar results, ^*^P<0.05 by t test.

**Figure 7:** JAK2/STAT3 functions in miR-216a inhibited EMT process and metastasis of GC cells **(A)** MGC-803 cells that were transfected with corresponding vectors were subjected to immunoblotting for JAK2, p-STAT3, STAT3, E-cadherin, N-cadherin and Vimentin. n = three repeats with similar results, ^*^P<0.05 by ANOVA. **(B)** JAK2 re-expression abolished the inhibitory effect of miR-216a on migration of MGC-803 cells. n = three repeats with similar results, ^*^P<0.05 by ANOVA. **(C)** JAK2 restoration facilitated invasion of miR-216a overexpressing MGC-803 cells. n = three repeats with similar results, ^*^P<0.05 by ANOVA.

**Figure 8:** The JAK2 inhibitor SAR317461 reverses the effects of miR-216a knockdown in GC cells **(A)** SGC-7901 cells that were transfected with miR-216a inhibitors (anti-miR-216a) were treated with the JAK2 inhibitor SAR317461 and DMSO, respectively. Western blotting data showed that SAR317461 treatment reduced the level of phosphorylated STAT3 and inhibited EMT process of SGC-7901 cells. n = three repeats with similar results, ^*^P<0.05 by t test. **(B)** SAR317461 treatment abrogated the promoting effect of miR-216a knockdown on migration of SGC-7901 cells. n = three repeats with similar results, ^*^P<0.05 by t test. **(C)** SAR317461 treatment restrained invasion of miR-216a silenced SGC-7901 cells. n = three repeats with similar results, ^*^P<0.05 by t test.

## DISCUSSION

Previous data demonstrate that miR-216a is involved in tumor initiation and progression, and its underexpression contributes to poor clinical outcome and cellular malignant phenotypes of CRC, pancreatic cancer, glioma and oral squamous cell carcinoma [10-13, 17]. Overexpression of miR-216a facilitates EMT and subsequently promotes metastatic behaviors of HCC and ovarian cancer cells [14, 15]. However, the clinical significance and biological function of miR-216a in GC were poorly investigated. Here, Our results showed that the levels of miR-216a were significantly lower in GC tissues compared to matched noncancerous tissues. Moreover, we disclosed that the expressions of miR-216a were reduced in GC cell lines. Clinical analysis revealed that miR-216a expression was an independent prognostic factor for predicting poor clinical outcome of GC patients. The mechanisms underlying the aberrant expression of miR-216a in human cancer is largely unknown. Previous study reports that miR-216a expression is upregulated by by the androgen pathway in a ligand-dependent manner in HCC [18]. Hypoxia, lncRNAs and methylation et al. have been implicated in regulation of miRNA expression [19–22]. Thus, the underlying mechanisms responsible for miR-216a underexpression require further investigation. Furthermore, low expression of miR-216a correlated with poor prognostic features and conferred a reduced survival in GC patients. Functionally, we demonstrated that miR-216a suppressed migration, invasion and EMT process of GC cells *in vitro* and *in vivo*. These data suggest that miR-216a exhibits an anti-metastatic role in the development of GC.

Previous studies showed that miRNAs regulated carcinogenesis by targeting its downstream molecules [23, 24]. Thus, predicting and confirming the targets of miR-216a are important to disclose the molecular mechanisms by which miR-216a suppressed metastasis of GC. In this study, JAK2 was identified as a direct target gene of miR-216a in GC cells by a luciferase reporter assay, which was consistent with the results in pancreatic cancer [13]. JAK2 is a member of the JAK family of protein tyrosine kinases, which performs diverse functional roles in carcinogenesis [25]. Previous studies suggest that JAK2 acts as an oncogene by regulation of phosphorylation of STAT3 in human HCC, lung cancer, CRC, pancreatic cancer and GC [26–30]. JAK2/STAT3 pathway plays a critical role in metastasis and EMT of GC cells [31, 32]. Therefore, it is valuable to study the regulatory effects of miR-216a in EMT process and metastasis of GC cells. Our results demonstrated miR-216a inversely modulated activation of JAK2/STAT3 pathway and the expressions of its downstream targets including Slug, Snail and Twist in GC cells. Slug, Snail and Twist are key regulator of EMT process in human GC [33–35]. Thus, we hypothesized that miR-216a inhibited EMT process and metastasis of GC cells probably by targeting JAK2/STAT3 pathway. Accordingly, we demonstrated that JAK2 restoration abrogated the anti-metastatic effects of miR-216a on GC cells with enhanced migration, invasion and EMT progression. These data solidly support our above hypothesis.

In conclusion, we demonstrate that the expression of miR-216a is restrained in GC tissues and cell lines. miR-216a underexpression associates with malignant clinical features and poor prognosis of GC patients. miR-216a inhibits migration, invasion and EMT process of GC cells probably by inhibiting activation of JAK2/STAT3 pathway. These findings suggest that miR-216a potentially plays an anti-metastatic role GC by targeting JAK2/STAT3 pathway.

## MATERIALS AND METHODS

### Human tissue samples, cell culture and transfection

Patients admitted to the China-Japan Union Hospital of Jilin University between January 2009 and December 2011 were evaluated. The study was approved by the Research Ethics Committee of the China-Japan Union Hospital of Jilin University, and all participants provided written informed consent. Diagnosis of GC was performed according to the criteria set by the American Joint Committee on Cancer (AJCC) staging system (6^th^ edition). Specimens including GC tissues and matched normal tissues from 90 patients were selected and pathologically diagnosed by experienced pathologists.

A normal human gastric epithelium cell line (GES-1) and GC cell lines (SGC-7901, MGC-803, MKN-28, and BGC-823) were purchased from the Institute of Biochemistry and Cell Biology, Chinese Academy of Sciences, Shanghai, China. Cells were cultured in the DMEM (Dulbecco’s modified Eagle’s medium) supplemented with 10% FBS (fetal bovine serum) in a humidified containing of 5% CO2 incubator at 37°C. Precursor miR-216a clones, miR-216a inhibitors and scrambled controls clones were purchased from Genecopoeia (Guangzhou, China). JAK2 overexpression vector and empty vector (EV) were obtained from Shanghai Genechem Co., LTD. (Shanghai, China). Cells were transfected using the Lipofectamine 2000 kit (Invitrogen, Carlsbad, CA, USA) according to the manufacturer’s instructions. The JAK2 inhibitor SAR317461 was obtained from (Sanofi-Aventis, Paris, France).

### Quantitative real-time polymerase chain reaction (qRT-PCR)

Total RNA was extracted from the GC tissues and cells using TRIzol reagent (Invitrogen) according to the manufacturer’s instructions [36]. Reverse transcription was performed using One Step PrimeScript miRNA cDNA Synthesis Kit (Takara, Dalian, China) following the manufacturer’s instructions. qRT-PCR was performed on an iCycler iQ™ Real-Time PCR Detection System (Bio-Rad Laboratories, Hercules, CA, USA). Primers for miR-216a and JAK2 were purchased from GeneCopoeia Co., (Guangzhou, China) Small nuclear RNA U6 and GAPDH mRNA were used as internal controls for calculating the relative expression levels of miR-216a and JAK2 via the 2^-ΔΔCt^ method.

### Western blot analysis

The transfected cells were lysed by RIPA lysis buffer (Beyotime, Jiangsu, China) for total protein extracts, and protein concentrations were measured following the BCA method (Beyotime). Cell lysates (30 μg/lane)were separated via sodium dodecyl sulfate polyacrylamide gel electrophoresis (SDS-PAGE). After being transferred to polyvinylidene fluoride membranes (Millipore, MA, USA), the proteins were incubated with primary antibodies against JAK2 (Cell Signaling Technology, Beverly, MA, USA), E-cadherin (Abcam, Cambridge, MA, USA), N-cadherin (Abcam), Vimentin (Abcam), p-STAT3 (Tyr705; Cell Signaling Technology), STAT3 (Cell Signaling Technology), Slug (Abcam), Snail (Abcam), Twist (Abcam) or GAPDH (Sigma, Santa Clara, CA, USA) at 4°C overnight, and further incubated in HRP-linked secondary antibodies (Santa Cruz Biotechnology, CA, USA) for 1 h at room temperature. Alpha Innotech (San Leandro, CA, USA) imaging software was used to quantify western blotting data.

### Immunofluorescence (IF)

GC cells that were transfected with corresponding miRNA vectors were seeded on chamber slides and fixed with 4% paraformaldehyde for 10 minutes at room temperature. Then, cells were incubated with primary antibodies including E-cadherin (Abcam) and Vimentin (Abcam) at 4°C overnight. Then, the slides were incubated with matched secondary antibodies (Invitrogen) at room temperature for 1 hour. The nuclear of EC cells were stained with DAPI (Sigma) at room temperature for 10 minutes. Fluorescence confocal images were captured using a LSM 5 Pascal Laser Scanning Microscope (Zeiss Germany, Oberkochen, Germany).

### Luciferase reporter assay

A fragment of the wild type (wt) JAK2 3′-UTR and a mutated (mt) JAK2 3′-UTR were cloned into the downstream region of the luciferase gene in the pGL3- REPORT luciferase vector (Invitrogen). For the luciferase assay, MGC-803 cells were co-transfected with pGL3-wt JAK2 3′-UTR or pGL3-mt JAK2 3′-UTR and precursor miR-216a or scrambled controls. Reporter activity was measured using a dual-luciferase reporter assay system (Promega, Madison, Wisconsin, USA). Firefly luciferase activity was normalized against Renilla luciferase activity.

### Migration and invasion assay

Wound healing assay was conducted by using Wound Healing culture inserts (Ibidi, Munich, Germany) following the manufacturer’s instructions. Wound closure rate was calculated to represent the cell migration ability. Cell invasion ability *in vitro* was assessed by using Matrigel-coated transwell inserts (BD Biosciences, Franklin Lakes, NJ, USA) following the manufacturer’s instructions. Cells invaded to the opposite side the membranes were counted.

### Experimental mouse model

BALB/c nude mice aged 4 week old were subjected to liver metastasis model. MGC-803 cells that were transfected with precursor miR-216a or scrambled controls were injected through the tail vein of nude mice and cultivated for 9 weeks. After euthanasia, the livers were harvested and fixed, paraffin-embedded, sectioned and stained for H&E [37], and the metastatic nodules were counted. All animal experiments were approved by the Ethics Committee of Harbin Medical University Cancer Hospital.

### Immunohistochemistry (IHC)

The tissues that were previously formalin-fixed and paraffin-embedded were sliced into 4 μm sections, and underwent deparaffination and then rehydration. Antigen retrieval, suppression of endogenous peroxidase activity and 10% skim milk blocking were performed before primary antibody incubation. JAK2 (Cell Signaling Technology) antibody was used as a primary antibody overnight at 4°C. The slides were subsequently incubated with peroxidase conjugated secondary antibody (ZSGB BIO, Beijing China) for 90 min, and a peroxidase-labeled polymer, DAB solution was used for signal development for 5 min. The sections were counterstained with hematoxylin followed by dehydrating and mounting. Staining intensity was scored as no staining = 0, weak staining = 1, moderate staining = 2, and strong staining = 3. Staining quantity was graded as <25% = 1, 25%-75% = 2, and >75% = 3. IHC score was manually confirmed by two independent experienced pathologists using the formula: IHC score = staining intensity × staining quantity.

### Statistical analysis

Data for continuous variables were presented as median ± standard deviation of data obtained from at least three independent experiments, and analyzed by GraphPad Prism 5 software (GraphPad Software, Inc, San Diego, CA, USA). Differences between groups were analyzed using Chi-squared test, student’s t-test or one-way ANOVA. Survival analysis was performed using Kaplan-Meier’s method and Log-rank test. Correlation analysis was analyzed by Spearman’s rank correlation test. P<0.05 was considered statistically significant.
